The article "ANS Responses and Facial Expressions Differentiate between the Taste of Commercial Breakfast Drinks" was published in 2014. Journal: PLoS One.

# ANS Responses and Facial Expressions Differentiate between the Taste of Commercial Breakfast Drinks

**DOI:** 10.1371/journal.pone.0093823

**Published:** 2014-04-08

**Authors:** René A. de Wijk, Wei He, Manon G. J. Mensink, Rob H. G. Verhoeven, Cees de Graaf

**Affiliations:** 1 Food and Biobased Research, Wageningen University and Research Centre, Wageningen, The Netherlands; 2 Division of Human Nutrition, Wageningen University, Wageningen, The Netherlands; Duke University, United States of America

## Abstract

The high failure rate of new market introductions, despite initial successful testing with traditional sensory and consumer tests, necessitates the development of other tests. This study explored the ability of selected physiological and behavioral measures of the autonomic nervous system (ANS) to distinguish between repeated exposures to foods from a single category (breakfast drinks) and with similar liking ratings. In this within-subject study 19 healthy young adults sipped from five breakfast drinks, each presented five times, while ANS responses (heart rate, skin conductance response and skin temperature), facial expressions, liking, and intensities were recorded. The results showed that liking was associated with increased heart rate and skin temperature, and more neutral facial expressions. Intensity was associated with reduced heart rate and skin temperature, more neutral expressions and more negative expressions of sadness, anger and surprise. Strongest associations with liking were found after 1 second of tasting, whereas strongest associations with intensity were found after 2 seconds of tasting. Future studies should verify the contribution of the additional information to the prediction of market success.

## Introduction

The high failure rate of new market introductions, despite initial successful testing with traditional sensory and consumer tests, necessitates the development of other tests. The low predictive validity of traditional sensory and consumer tests, which include sensory analytical profiling and liking tests, may be due to the fact that these tests require cognitive information processing and rational reasoning whereas consumer behavior may be more based on unarticulated/unconscious motives and associations. Reasons for food choice include sensory affective reasons (dislike/like of the food), but also anticipated consequences of ingestion (satiation, illness) and ideational reasons (knowledge of the nature or origin of the food) [1]. In addition, food pleasure and food choice also depends on the simultaneous internal context (food choice in a hungry state will be different from that in a satiated state), simultaneous external factors (food choice will be affected when informed that the food may be spoiled), and successive external context (pleasure of food decreases during consumption whereas pleasure of non-consumed food is unaffected, a phenomenon also known as sensory-specific satiety [2]).

The article "ANS Responses and Facial Expressions Differentiate between the Taste of Commercial Breakfast Drinks" was published in 2014. Journal: PLoS One.

The combined effect of these factors on food choice is mediated by emotional responses, such as disgust when one is informed that the consumed food was spoiled. Frijda [3] distinguishes the following elements of emotions: *affect*, or the hedonic pleasure of foods, *appraisal* of foods in terms of good/bad or pleasant/unpleasant, *action readiness* (whether or not the food is consumed), and *autonomic arousal* reflecting the degree of motor preparation for the action. Affect and appraisal are typically assessed explicitly via questionnaires (e.g. [4], [5] or implicitly via facial expressions (e.g. [6]–[10]). Action readiness and autonomic arousal are typically assessed implicitly with physiological measures of the autonomic nervous system (ANS, see also [11]). More recently, the notion was introduced that various aspects of stimuli are appraised sequentially [12] whereby each type of appraisal is associated with specific physiological, expressive and motivational changes. For example, Aue and colleagues (2007) [13] presented participants with pictures that displayed biological and cultural threats or neutral stimuli, and demonstrated with EEG and facial muscle activity that relevance appraisal preceded goal conduciveness appraisal. Similarly, Delplanque and colleagues [14], using facial muscle activity and electrodermal activity and olfactory stimuli, demonstrated that novelty reactions precede pleasantness reactions. In one of the few food studies in which responses from the autonomic nervous system (ANS) were recorded, De Wijk et al [15] demonstrated that ANS responses differentiated between the sight of foods that were liked and disliked. Moreover, ANS responses to the sight of a food varied with the instruction to either view, smell or taste the food. ANS responses to the taste of the foods were not measured in that study.

ANS responses and facial expressions to the taste of foods were recorded in the present study. Unlike the previous study, foods with a single product category (breakfast drinks) with similar valence were used in this study. Moreover, responses were monitored continuously during tasting to allow testing of sequential appraisals. The study tested whether:

- ANS responses and facial expressions discriminated between foods with similar valence.
- Liking and intensity are associated with different response patterns and with different response times.

The article "ANS Responses and Facial Expressions Differentiate between the Taste of Commercial Breakfast Drinks" was published in 2014. Journal: PLoS One.

## Methods

### Participants

Nineteen adults (10 females; mean age 30.1±11.7 years and 9 males, mean age 36.2±12.7 years) were tested. The study was approved by the Medical Ethical Committee of the Wageningen University. Participants were recruited from the subject pool of the Consumer Science and Intelligent Systems department of the Wageningen University. All participants signed an informed consent form and received an incentive for their participation.

### Breakfast Drinks

Five commercially available breakfast drinks were used for the study. The breakfast drinks included three drink yoghurts (Royal Friesland Campina), Goede Morgen fruit Aardbei-kiwi-banaan (GM Str), Goede Morgen original Perzik-abrikoos (GM Pea) and Goede Morgen fruit Sinaasappel-mango-banaan (GM Sin), and two fruit drinks (Hero): Fruit Ontbijt original Bosvruchten (FO BV) and Fruit Ontbijt original Sinaasappel-banaan (FO Sin). A sixth commercial breakfast drink was used once as a warm-up sample at the beginning of a session. The drinks were presented to the participants in 250 ml glasses. Drinking straws were used by participants to sample from each drink because normal drinking would cause severe visual artefacts in the facial expressions and motor artefacts for the ANS responses. Participants took a single sip from each drink. Based on an estimated sip size of 10 ml, participants consumed on average a total of 250 ml during a session.

### Design

In the experimental session the five breakfast drinks were presented in five blocks of five food presentations. Each drink was presented once per block in a randomized order. The presentations were separated by an interval of 60 seconds. Within-subjects designs with five outcome measures (skin conductance response (SCR), heart rate frequency (HR), skin temperature (ST), facial expressions, and ratings) were used. A sixth presentation was included in the study where participants rated their emotional responses to each of the drinks. These results will be reported separately.

### Physiological ANS Measures

Physiological measures included:

1. Skin conductance response or SCR measured in μSiemens with electrodes placed on the palm of the non-dominant hand of the participant;
2. Heart rate or HR measured in beats per minute with electrodes placed on the chest;
3. Skin temperature or ST measured in Celsius degrees with an electrode placed on the palm of the non-dominant hand of the participant.

The physiological data were collected via a Mindware Acquisition data acquisition system (Mindware Technologies, Inc.) with separate filter settings for the electrocardiogram, skin temperature and electrodermal (skin conductance response) activity. Filter settings were low-pass 0.5 Hz, high-pass 45 Hz for heart rate frequency, low-pass 1 Hz, high-pass 45 Hz for SCR and low-pass 10 Hz, high-pass 45 Hz for skin temperature. Electrodes were used with a surface of 4.1 cm and filled with 1% Chloride wet gel. Signals were transferred to the Acquisition Unit (16 bit A/D conversion) and stored on computer hard disk (sampling rate 500 Hz/s). Electrocardiographic R waves were detected offline, and intervals between heartbeats were converted to heart rate, expressed in beats per minute (BPM). SCR activity was recorded (high-pass filter: 0.025 Hz.) by the constant voltage method (0.5 V). The signal was amplified by 1,000 and low-pass filtered (30 Hz). SCRs were analysed off-line after correction for baseline.

The article "ANS Responses and Facial Expressions Differentiate between the Taste of Commercial Breakfast Drinks" was published in 2014. Journal: PLoS One.

### Behavioral Measures

Facial expressions were automatically analyzed using FaceReader software version 4.0 (Noldus Information Technology, Wageningen, The Netherlands). FaceReader works in three steps: 1) face finding, 2) face modelling, and 3) face classification. During face finding an accurate position of the face is found using the Active Template Method. During modelling, the Active Appearance Model is used to synthesize an artificial face model, which describes the location of 491 key points as well as the texture of the face. The actual classification of the facial expressions is done by training an artificial neural network as training material nearly 2000 manually annotated images were used. The network was trained to classify the six basic or universal emotions described by Ekman [16]: happy, sad, angry, surprised, scared, and disgusted and a neutral state. FaceReader analyzed the facial expressions on a frame by frame basis, i.e. at 25 Hz.

### Liking and Intensity Scores

Liking and overall intensity was rated on visual analog scales of 10 cm length. The liking scale was anchored “absolutely unpleasant” on the left side and “absolutely pleasant” on the right side. The intensity scale was anchored “very low intensity” on the left side and “very high intensity” on the right side.

### Procedure

#### Instruction and set-up

The experimental sessions took place in the physiological laboratory of the Restaurant of the Future located in Wageningen, the Netherlands. The experiment leader explained the experiment to the participant, allowed ample time for questions and asked the participant to sign the inform consent form (which they had received by e-mail prior to the experimental session) after which the electrodes were placed. A camera placed about one meter in front of the participant to measure the facial expressions was adjusted in height to get a clear view of the face of the participant. The camera was placed just above a computer monitor that was used to instruct the participant. A second camera was placed on the right side of the participant to identify the exact moment of tasting. The seat of the participant was also adjusted if necessary. The breakfast drinks were prepared in transparent 250-ml drinking glasses with a drinking straw normally placed outside the viewing area of the participant. The participants were instructed to look straight in the direction of the camera. Oral instructions were given by the experiment leader. The instructions were manually timed by a researcher to allow the participants enough time to taste the presented food product. After the instruction, participants received a practice trial with a breakfast drink that was not used in the rest of the study. Next, the experimental measurements started where participants received a number of trials. Per trial, one breakfast drink was presented.

The article "ANS Responses and Facial Expressions Differentiate between the Taste of Commercial Breakfast Drinks" was published in 2014. Journal: PLoS One.

#### Trial

A session consists of a series of trials. During each trial, participants sipped from one of the breakfast drinks. The trial procedure was developed to minimize unwanted motor artefact that may affect the physiological measurements and to provide optimal conditions for the FaceReader automated expression analysis. Each trial started with an auditory attention signal to indicate that the participant had to look in the direction of the camera and the computer monitor, and that the trial was about to start. For 10 seconds a photograph of the breakfast drink in a glass cup was shown on the monitor to mimic the normal situation where one sees the drink before tasting. Simultaneously, a glass with the same breakfast drink plus straw was put near the participants head. After 10 seconds the photo was replaced by the instruction to take the straw in the mouth but not drink, which was replaced after 6 seconds by the instruction to take a sip and to leave the straw in the mouth. After 10 seconds the participant was instructed to remove the straw and to enter the liking and intensity of the breakfast drink using 10 point rating scales (see also Figure 1). Before the next trial the researcher removed the cup. The physiological and behavioral measures were continuously recorded.

**Figure 1:** Scheme of experiment procedures.

### Data Analysis

The processed images with the facial expressions were combined with the images from the other camera, and with raw physiological data combined in Observer XT 10.5 software (Noldus Information Technology, Wageningen, The Netherlands) for further analyses. Markers were placed manually to identify the moments of the participant’s first visual contact with the drink and of the first sip. Only the results for the first sip will be reported here.

The article "ANS Responses and Facial Expressions Differentiate between the Taste of Commercial Breakfast Drinks" was published in 2014. Journal: PLoS One.

#### Physiological measures

The physiological measures skin conductance response (SCR), heart rate (HR) and skin temperature (ST) were analyzed per experimental session. SCRs were measured in μSiemens, analyzed offline, and corrected for baseline. ST was expressed as change in temperature over the 10 seconds relative to the temperature at t = 0.

#### Facial expressions

The video images of the facial expressions were processed with FaceReader 4.0 software (Noldus Information Technology, Wageningen, The Netherlands) which determined the facial micro-expressions based on Active Appearance Modelling [17] in each time frame (at a frequency of 25 Hz) during 10 seconds after tasting. A more detailed description of the science behind FaceReader can be found at: http://info.noldus.com/free-white-paper-on-facereader-methodology/.

#### Statistical analysis

Inspection of the ANS results and facial expressions indicated largest effects during the first five seconds of tasting. Mixed model ANOVAs were carried out with participants as random factor and time (1–5 seconds), gender, breakfast drink and replicate as fixed factors (IBM SPSS statistics, version 19). Partial Least Square analysis (Unscrambler, CAMO ASA, Oslo, Norway) was used to evaluate associations between facial expressions and ANS measures during 0.25 second intervals after stimulation with valence and intensity of the drinks (reflected by liking and intensity ratings). Correlation coefficients between observed and predicted liking or intensity values were used as indicator for the strength of associations, and regression coefficients were used to identify the facial expression that contribute most to these associations.

## Results

### Physiological Measurements

#### Skin temperature

Changes in skin temperature vary significantly with gender, drink, and replicate. Replicate affected changes in skin temperature drink with replicate were drink-specific (drink × rep interaction) (see Table 1, and Figure 2A). All main effects and interactions varied with gender.

**Figure 2:** Changes in ANS measures during tasting of five breakfast drinks. Results of Skin temperature (**A**), Heart rate (**B**), and Skin conductance response (**C**) are averaged across participants and replicates.

**Table 1:** Output of mixed model ANOVAs carried out on physiological ANS measures and facial expressions with participants as random factor, and gender (M/F), replicate (1–5), drink (1–5), and time (1–5 seconds) as fixed factors.

	Physiological measures							Facial expressions														
		Heart rate		Skin conductance		Skin temperature			Neutral		Happy		Angry		Sad		Surprised		Scared		Disgusted	
	d.f.	F	p	F	p	F	p	d.f.	F	p	F	p	F	P	F	p	F	p	F	p	F	p
**Gender**	1,1591	96.9	0.001	168.1	0.001	83.1	0.001	1,1882	130.2	0.001	61.3	0.001	110.2	0.001	184.5	0.001	0.03	ns	56.8	0.001	19.4	0.001
**Rep**	1,1591	2	ns	0	ns	21.8	0.001	1,1882	2	ns	2.9	0.02	7.7	0.001	1.6	ns	10.8	0.001	5.1	0.001	1.4	ns
**Drink**	4,1591	63.3	0.001	0	ns	4.1	0.003	4,1882	0.2	ns	3.1	0.01	0.7	ns	0.8	ns	0.7	ns	1.5	ns	1.2	ns
**Time**	4,1591	12.5	0.001	1.1	ns	0.2	ns	4,1882	3.3	0.01	1.7	ns	1.4	ns	0.8	ns	0.9	ns	5.8	0.001	2.2	ns
Gender*Rep	4,1591	3.7	0.005	0.1	ns	5.2	0.001	4,1882	4.1	0.003	5.4	0.001	7.8	0.001	1.3	ns	1.9	ns	1.8	ns	1.5	ns
Gender*Drink	4,1591	2.9	0.02	0.1	ns	5.5	0.001	4,1882	1.6	ns	4.9	0.001	0.1	ns	3.2	0.01	0.4	ns	0.3	ns	0.7	ns
Gender*Time	4,1591	0.4	ns	0.4	ns	1.4	ns	4,1882	5.1	0.001	2.3	ns	1.7	ns	4.1	0.002	3	0.02	4.6	0.001	1.4	ns
Rep*Drink	16,1591	0.3	ns	0	ns	8.9	0.001	16,1882	0.2	ns	0.5	ns	0.1	ns	0.3	ns	0.3	ns	0.4	ns	0.5	ns
Rep*Time	16,1591	1.5	ns	0.1	ns	0.6	ns	16,1882	1.2	ns	1.4	ns	1.6	0.05	2.4	0.001	2	0.01	3.1	0.001	2.3	0.003
Drink*Time	16,1591	0.2	ns	0	ns	0.3	ns	16,1882	0.2	ns	0.3	ns	0.3	ns	0.2	ns	0.9	ns	0.2	ns	0.3	ns
Gender*Rep*Drink	16,1591	0.1	ns	0	ns	4.4	0.001	16,1882	0.3	ns	0.1	ns	0.2	ns	0.38	ns	0.6	ns	0.2	ns	0.2	ns
Gender*Rep*Time	16,1591	0.6	ns	0.2	ns	0.2	ns	16,1882	2.9	0.001	1	ns	1.9	0.02	2.2	0.004	3.3	0.001	2.7	0.001	4.3	0.001
Gender*Drink*Time	16,1591	0.3	ns	0	ns	0.2	ns	16,1882	0.1	ns	0.3	ns	0.2	ns	0.1	ns	0.6	ns	0.2	ns	0.2	ns
Rep*Drink*Time	64,1591	0.2	ns	0	ns	0.2	ns	64,1882	0.2	ns	0.2	ns	0.1	ns	0.2	ns	0.5	ns	0.3	ns	0.2	ns

The article "ANS Responses and Facial Expressions Differentiate between the Taste of Commercial Breakfast Drinks" was published in 2014. Journal: PLoS One.

#### Heart rate

Heart rates increase during the first seconds of tasting followed by a gradual decrease. Heart rate frequency varies significantly with drink (see Table 1, and Figure 2B). Gender affected heart rate both as main effect and in interaction with drink, replicate and time.

#### Skin conductance responses

Instead of the expected rise and subsequent decline of SCR during tasting, only decline is observed in this study. Skin conductance responses are not affected significantly by drink or replicate (see Table 1 and Figure 2C).

### Facial Expressions

The temporal development of facial expressions during tasting is summarized in Figure 3 based on the averaged values across drinks and replicates. Some expressions such as happiness, neutral, and surprise show an initial increase after tasting that reaches a maximum at intervals between 0.5 second (surprise) and 4 seconds (happiness). In contrast, expressions of disgust continue to increase over at least 7 seconds. Other expressions such as sadness, scared, and angry show an initial decrease that reaches a minimum between 1.5 (sadness) and 3 seconds (scared). The initial increase or decrease is either followed by a return to baseline (sadness, scared, surprised), a decrease (happiness, neutral) or an increase (angry).

The article "ANS Responses and Facial Expressions Differentiate between the Taste of Commercial Breakfast Drinks" was published in 2014. Journal: PLoS One.

**Figure 3:** Facial expressions averaged across participants, breakfast drinks and replicates, during 10 seconds of tasting.

All facial expressions varied with drink, either as main effect (neutral, happy, angry, surprised and scared) and/or in interaction with time (angry, surprised, scared, sad and disgust). Neutral, happy and sad expressions varied with replicate either as main effect (happy) or in interaction with the participant’s gender (neutral and sad). All expressions, except surprise, varied significant with gender (see Table 1).

### Liking and Intensity

Liking scores did not vary with breakfast drinks, replicate or their interaction (see Table 2). Intensities did vary with breakfast drink (F(5,31) = 2.6, p = 0.04), replicate (F(1,31) = 5.8, p = 0.02) and their interaction (F(5,31) = 3.5, p<0.01 (see Table 3).

**Table 2:** Liking scores (SD) per breakfast drink and replicate averaged across participants.

Liking	FO sinas.-banaan	FO Bos vruchten	GM Perzik-abrikoos	GM Sinaasappel-mango-banaan	GM Aardbei-kiwi-banaan
**Replicate 1**	5.8 (1.8)	5.0 (1.9)	5.9 (1.4)	5.9 (1.4)	6.1 (1.6)
**Replicate 2**	5.4 (1.8)	5.3 (2.0)	5.6 (1.5)	5.5 (1.4)	6.5 (1.2)
**Replicate 3**	5.3 (1.7)	5.3 (1.9)	5.6 (1.3)	5.5 (1.5)	5.9 (1.5)
**Replicate 4**	5.3 (1.7)	5.0 (1.6)	5.1 (1.7)	5.4 (1.4)	6.2 (1.8)
**Replicate 5**	5.7 (2.0)	4.7 (1.8)	5.0 (2.2)	5.5 (1.8)	6.2 (1.4)

**Table 3:** Intensity scores (SD) per breakfast drink and replicate averaged across participants.

Intensity	FO sinas.-banaan	FO Bos vruchten	GM Perzik-abrikoos	GM Sinaasappel-mango-banaan	GM Aardbei-kiwi-banaan
**Replicate 1**	6.0 (1.0)	5.4 (1.4)	6.0 (0.9)	6.1 (1.1)	5.7 (1.6)
**Replicate 2**	6.4 (1.5)	5.7 (1.2)	5.4 (1.3)	6.2 (1.0)	6.3 (1.0
**Replicate 3**	6.4 (1.2)	6.2 (1.2)	5.6 (1.0)	6.2 (1.3)	5.9 (1.4)
**Replicate 4**	6.4 (1.2)	6.4 (1.2)	5.6 (1.1)	6.0 (1.0)	6.2 (1.1)
**Replicate 5**	6.8 (0.9)	6.4 (1.4)	6.0 (1.5)	6.0 (1.3)	5.7 (1.2)

### Liking and Intensity Scores Versus other Measures

Despite the fact that liking scores did not vary systematically between drinks and/or replicates, they still showed some variation (between 4.7 and 6.5 on a 10 point ratings scale). Partial least square analysis was used to verify systematic relations between liking scores and physiological measurements and facial expressions at various intervals during tasting. The degree of correspondence between the observed liking scores and the ones predicted from the PLS models, expressed by correlation coefficients, gradually decreased from 0.51 (after 1 second of tasting) to 0.39 and 0.47 (respectively after 3 and 4 seconds of tasting) (critical correlation coefficient (p = 0.05) is 0.40 (n = 25). The contribution of facial expressions and ANS measures to liking was reflected by the PLS regression coefficients shown in Figure 4A. Liking scores were positively associated with increased heart rate, skin temperature, to a lesser degree with increased skin conductance, and with neutral facial expressions. Liking scores were negative associated with all other facial expressions, including those of happiness.

The article "ANS Responses and Facial Expressions Differentiate between the Taste of Commercial Breakfast Drinks" was published in 2014. Journal: PLoS One.

**Figure 4:** Regression coefficients from the partial least squares analysis . ANS measures and facial expressions during 1–4 seconds of tasting are dependent variables. Liking (**A**) or intensity (**B**) is independent variables.

Liking scores were best predicted from facial expressions during the first replicate, i.e., the observed and predicted liking scores were most similar for the first replicate. During subsequent replicates the average deviation between observed and predicted liking scores grew from 2% (replicate 1) to 9% (replicate 5).

The degree of correspondence between the observed intensity scores and the ones predicted from the PLS models grows from 0.47 for the first second to 0.62 for the second second after which it gradually decreases to 0.55 for the fourth second (critical correlation coefficient (p = 0.05) is 0.40 (n = 25). Intensity scores were negatively associated with skin temperature and to a lesser degree with heart rate, and with expressions of happiness, disgust, and scared. Intensity scores were positively associated with skin conductance, and with expressions of neutral, surprise, sad and anger (see Figure 4B).

Similar to liking scores, intensity scores were best predicted from facial expressions during the first replicate. During subsequent replicates the average deviation between observed and predicted intensity scores grew from 2% (replicate 1) to 5% (replicate 5).

## Discussion

The study used facial expressions and ANS responses to verify systematic differences between similar and well-liked breakfast drinks, and to explore associations with liking and intensity. Whereas liking scores, the traditional sensory tool to measure product “performance”, failed to show systematic differences between drinks and/or replicates, physiological ANS measures and facial expressions were sensitive enough to demonstrate differences between drinks and between replicates. The relevance of the differences between liking results and ANS/facial expression results is unclear. Liking scores are probably not the gold standard for the prediction of success of new market introductions because most new food introductions disappear from the market despite high liking scores in prior sensory and marketing tests. Whether ANS/facial expression results offer better predictions remains to be tested, for example with exact sales data per drink. Unfortunately, sales data are typically not available to researchers.

The article "ANS Responses and Facial Expressions Differentiate between the Taste of Commercial Breakfast Drinks" was published in 2014. Journal: PLoS One.

ANS responses and facial expressions proved to be highly dynamical over time with specific time courses for each measure. Heart rate initially increased followed by a decrease, skin temperature either increased or decreased dependent on the breakfast drink, whereas skin conductance typically decreased. Facial expressions proved to be even more dynamical both in terms of their time course and in their magnitude. Early facial expressions are for example dominated by neutral and surprise whereas later expressions are dominated by disgust. The dynamical nature of the responses may be related to their association with liking and intensity; relatively early responses (after approximately 1 second of tasting) show strongest associations with liking scores obtained afterwards whereas somewhat later responses (after approximately 2 seconds) showed strongest associations with intensity scores. These results suggest that different aspects of the stimuli are processed – or appraised- at different times. These results are in line with results from other studies showing for example that relevance appraisal precedes goal conduciveness appraisal [13] and novelty appraisal precedes pleasantness appraisal [14] providing support for current models of emotions by Scherer and colleagues [12].

Liking was positively associated with neutral expressions and negatively associated with facial expressions of sadness, anger, surprise, and scared. This supports previous findings of Zeinstra et al. (2009) [10]who demonstrated that facial expressions reflected disliking but not liking of stimuli. Unexpectedly, liking and ANS parameters are also negatively associated with expressions of happiness, i.e., reduced liking is associated with more facial expressions of happiness. Facial expressions of happiness are rarely displayed when one is alone and social interactions are absent suggesting that these expressions serve a social function [18], [19]. The fact that they did occur in this study in the presence of experimental staff suggests that the happy facial expressions may serve some kind of social signaling function, e.g., to signal the staff that one is OK despite the previous display of for example negative expressions.

Liking was positively associated with heart rate and skin temperature which is in line with previous research that demonstrated a positive association between these ANS parameters and positive emotions of joy [11]. The positive association between heart rate and liking found for consumed foods in the present study contradicts previous findings for odors where odor pleasantness is typically inversely related to heart rate [20]. Kreibig’s review [11]already demonstrates that interpretation of patterns in ANS results is typically not straight-forward but dependent on factors such as task demands and stimulus modality. For example, our findings show that consumption of as little as one sip already increases heart rate by 10–14 beats/min, irrespective of the drink, whereas sniffing an odor led to much smaller increases for unpleasant odors (3–4 beats/min) and unchanged heart rates for pleasant odors [20]. These different patterns make a direct comparison of results across modalities difficult.

The article "ANS Responses and Facial Expressions Differentiate between the Taste of Commercial Breakfast Drinks" was published in 2014. Journal: PLoS One.

Very different associations were found for intensity scores. Higher intensities were associated with lower heart rate and skin temperature, patterns that had been associated by others to negative emotions of fear, disgust, sadness, anger and anxiety [11]. In the present study, higher intensities also resulted in more facial expressions signaling negative emotions such as sadness and anger, but also with more neutral and surprised expressions and fewer expressions of happiness, scared and disgust. Hence, facial expressions and ANS results are partly inconsistent in the case of intensities for unknown reasons.

Skin conductance and temperature responses suggest that participants not only respond to the actual taste of the breakfast drink but also to the preceding image of the product; the typical ascending phase followed by the descending phase of skin conductance responses is absent in our taste responses suggesting that participants already anticipated the taste during the preceding image of the drink. Similarly, skin temperatures already differ between breakfast drinks at the start of tasting suggesting pre-tasting effects of the preceding images. These pre-tasting effects should be weakest during the first replicate when image-taste associations are relatively new, and should grow stronger with each additional replicate. Indeed, our results demonstrate that facial expressions and ANS responses during tasting best predict liking and intensity for the first replicate and that predictions become poorer with additional replicates. We hypothesize that with stronger image-taste associations participants probably respond more and more to the image of the breakfast drink and less and less to the taste itself; i.e., they have learnt the expected taste from the images. According to this hypothesis, the association between facial expressions/ANS responses and intensity/liking should shift with increasing replicates from responses during tasting to responses during viewing, but this was not tested in this study. Pre-tasting anticipatory responses to visual food stimuli have been investigated previously before where it was demonstrated that facial expressions and ANS responses to visual foods reflected the anticipation of participants to either view, smell, or taste the foods [15].

The article "ANS Responses and Facial Expressions Differentiate between the Taste of Commercial Breakfast Drinks" was published in 2014. Journal: PLoS One.

Contributions to the prediction of market success may not be the only reason for selection of physiological measures and/or facial expressions. These measures offer advantages over other more traditional measures because they are relatively fast (typically a matter of seconds rather than minutes as required for questionnaires) which facilitates linkage to specific phases of product-consumer interactions. In addition, these measures may reflect processes that consumers are not even aware of, and that are therefore difficult to capture with questionnaires, but which may contribute to consumer decisions. On the other hand, facial responses and physiological measurements are technically more challenging than questionnaires and applications are therefore more suitable for laboratory than for real-life.

In conclusion: ANS measures and facial expressions differentiate between repeated exposures to members of a homogeneous group of well-liked breakfast drinks. Relatively fast responses show mostly differentiation based on liking, whereas somewhat later responses show mostly differentiation based on intensity. ANS responses and facial expressions may contribute to the development of new food products that are not only initially liked, but that are also liked over the long term.
